The article "An Expeditious Synthesis of [1,2]Isoxazolidin-5-ones and [1,2]Oxazin-6-ones from Functional Allyl Bromide Derivatives" was retracted in 2014. Reasons: misconduct by an author; duplicated images; duplicated data.

# An Expeditious Synthesis of [1,2]Isoxazolidin-5-ones and [1,2]Oxazin-6-ones from Functional Allyl Bromide Derivatives 

**DOI:** 10.3390/molecules15064094

**Published:** 2010-06-07

**Authors:** Imen Beltaïef, Aïcha Arfaoui, Hassen Amri

**Affiliations:** Laboratoire de Chimie Organique et Organométallique, Université de Tunis El Manar, Faculté des Sciences, Campus Universitaire 2092-Tunis, Tunisia

**Keywords:** functional allyl bromides, conjugate addition, *N*-substituted hydroxylamines, isoxazolidin-5-ones, oxazin-6-ones

## Abstract

Reaction of allyl bromide **(*Z*)-1 **and** (*Z*)-2 **with *N*-substituted hydroxylamine hydrochlorides in presence of *tert*-butoxide in *tert*-butanol at reflux provides a short and effective route to [1,2]isoxazolidin-5-ones **3** and [1,2]oxazin-6-ones **4**.

## 1. Introduction

Acrylic compounds have become highly attractive and building blocks for the synthesis of several biologically active molecules such as α-methylene-γ-butyrolactones [1,2,3,4,5] and γ-butyrolactams [6,7,8,9]. Several studies have proposed methods for the preparation of compounds bearing a α-bromomethyl moiety [10,11,12,13,14] commonly called Baylis-Hillman bromides [15,16,17,18,19]. In an ongoing project aimed at further illustrating the potential of readily prepared α-bromomethylated esters analogs **2** [9,20], we have shown the importance of functional allylic bromide **2** as an electrophilic reagent for access to pyrrolidin-2-ones [9], α-alkyl-β-carbomethoxy-γ-butyrolactams [21,22], (*E*,*Z*)-α-alkylidene-γ-butyro-lactones [23] and 4-methoxycarbonyl-1-*N*-alkyl-∆^2^-pyrrolidin-2-ones. In order to explore the potential of hydroxylamines in organic synthesis, we have been examining their nucleophilic reactivity as an *N*,*O*-centered tandem nucleophile. We report here a direct synthesis of isoxazolidin-5-ones **3** and oxazin-6-ones **4** *via* Michael addition then intramolecular cyclization of *N*-substituted hydroxylamines to functional allyl bromides (***Z***)-**1 **and (***Z***)-**2** (Scheme 1).

**Scheme 1:** Synthesis of [1,2]oxazin-6-ones and [1,2]isoxazolidin-5-ones from allyl bromides **1**-***Z*** and **2***-**Z***.

## 2. Results and Discussion

Despite the interesting potential synthetic and pharmacological value of the isoxazolidin-5-ones **3**, there are only a few works in the literature reporting their synthesis [24,25]. The majority of the recorded examples have been prepared by condensation of ester enolates and their equivalents [26,27,28,29] or pyrazolidinone acrylamides [30] with *N*-substituted hydroxylamines. More recently, α,β-sugar lactones [31,32,33] were used as good starting Michael acceptors to produce the isoxazolidin-5-one ring system, thus providing an effective route for the selective formation of substituted azetidin-2-ones [34,35] or β-substituted-β-amino acids [36]. In order to examine the feasibility of the route outlined in Scheme 2, available allyl bromides (***Z***)-**1** were prepared. Then, their condensation with a variety of *N*-substituted hydroxylamine hydrochlorides in the presence of potassium *tert*-butoxide in *tert*-butanol at reflux was carried out, which results in the formation of isoxazolidin-5-ones **3 **in good yields, as shown in Table 1. 

The article "An Expeditious Synthesis of [1,2]Isoxazolidin-5-ones and [1,2]Oxazin-6-ones from Functional Allyl Bromide Derivatives" was retracted in 2014. Reasons: misconduct by an author; duplicated images; duplicated data.

**Scheme 2:** Synthesis of (*E*)-4-alkylidene-2-alkylisoxazolidin-5-ones **3** from allyl bromide (***Z***)-**1**.

**Table 1:** (*E*)-4-Alkylidene-2-alkylisoxazolidin-5-ones **3a-e **prepared.

Product	R^1^	R^2^	Yield *^a^* (%)
**3a**	*^n^*C_3_H_7_	*^t^*C_4_H_9_	60
**3b**	C_6_H_5_	*^t^*C_4_H_9_	83
**3c**	*^n^*C_3_H_7_	*^c^*C_6_H_11_	48
**3d**	C_6_H_5_	*^c^*C_6_H_11_	61
**3e**	*^n^*C_5_H_11_	*^c^*C_6_H_11_	56

*^a^* Isolated yield after chromatography.

The initial reaction was considered to be, as described before in our previous work [37], a conjugated addition of the hydroxylamine amino group to the allyl bromide (***Z***)-**1 **leaving an ammonium intermediate which reacted with second hydroxylamine equivalent leading to an expected S_N_2 product followed by a reasonable transesterification (5-*exo-*trig process) to give (*E*)-4-alkylidene-2-alkylisoxazolidin-5-ones **3** as only isolated products in fair to good yields (48–83%) and with total (*E*)-stereoselectivity (Scheme 2, Table 1).

Although this route in fact proved a successful strategy to access to the five-membered ring heterocyclic system of [1,2]isoxazolidin-5-ones **3**, we considered the possibility of a more efficient and shorter sequence to generate uncommon six member structures bearing the *N-O* linkage, in particular [1,2]oxazin-6-ones **4**. Since the [1,2]oxazine and [1,2]oxazinone skeletons have recently been found to be the central features in antitumor and antibiotic products [38,39,40], synthetic methods providing access to these skeletons have gained considerable attention [41,42,43,44]. To the best of our knowledge, there are only a few literature reports on this topic [45,46,47]. As shown in Scheme 3, we found that the conjugate addition of *N*-substituted hydroxylamine hydrochlorides (3 equiv.) to dimethyl (*Z*)-2-(bromomethyl) fumarate (**2**) afforded pure [1,2]oxazin-6-ones **4 **in fair to good yields. 

**Scheme 3:** *N*-Substituted hydroxylamine addition to dimethyl (*Z*)-2-(bromomethyl) fumarate (**2**).

**Table 2:** Methyl 2-alkyl-6-oxo-5,6-dihydro-*2H*-1,2-oxazine-4-carboxylate **4a-e **prepared.

Product	R	Yield *^a^* (%)
**4a**	*^i^*C_3_H_7_	79
**4b**	*^t^*C_4_H_9_	76
**4c**	*^c^*C_6_H_11_	58
**4d**	C_6_H_5_	35
**4e**	CH_2_C_6_H_5_	6

*^a^* Isolated yield after chromatography.

The article "An Expeditious Synthesis of [1,2]Isoxazolidin-5-ones and [1,2]Oxazin-6-ones from Functional Allyl Bromide Derivatives" was retracted in 2014. Reasons: misconduct by an author; duplicated images; duplicated data.

The synthetic approach proceeds through a two-step sequence as expected: allylic substitution (S_N_2’) of allyl bromide **2** by the *N*,*O*-binucleophilic reagent providing a zwitterion cyclobutane intermediate whose opening leads to the most stable (*E*) enaminic structure, then a spontaneous 6-*exo*-trig [48] cyclization process, leading to the formation of **4**. Additional proof of the enaminic system in [1,2]oxazin-6-one **4a **came from the ^1^H- and ^13^C-NMR data, which unequivocally showed the high and low values of the shifts of the vinylic proton at 8.04 ppm and both allylic carbon atom at 27.1 ppm, respectively. Surprisingly, the chemical yields were notably lower when *N*-substituted hydroxylamine moieties bearing phenyl and benzyl groups were used; this is probably due to the low solubility of the intermediary imine in the *tert*-butanol solvent before cyclization. 

## 3. Experimental

### 3.1. General

All reactions were monitored by TLC on silica gel plates (Fluka Kieselgel 60 F_254_). For column chromatography, Fluka Kieselgel 70-230 mesh was used. ^1^H- and ^13^C-NMR spectra (fully decoupled) were recorded on a Bruker AMX 300 instrument in CDCl_3_ as solvent and with TMS as the internal standard. IR spectra were recorded with a Perkin-Elmer Paragon 1000 FT-IR spectrophotometer. Mass spectrometry was performed on an Autospec 200 Micromass instrument (Waters). Most of the reagents and solvents were obtained from commercial sources (Aldrich, Merck, Fluka) and used as received. Except for the commercially available dimethyl itaconate, allyl bromides **1** and **2** were prepared as described in references [16] and [8], respectively.

### 3.2. General procedure for the synthesis of (E)-4-alkylidene-2-alkylisoxazolidin-5-ones ***3***

*N*-Alkylhydroxylammonium chloride (30 mmol) and potassium *tert*-butoxide (28 mmol) in *tert*-butanol (45 mL) were placed in a 100 mL flask under a nitrogen atmosphere. The reaction mixture was stirred at reflux for 10 minutes then allyl bromide **1-*Z*** (10 mmol) was added. After the disappearance of the substrate (TLC), the mixture was filtered under reduced pressure, evaporated and purified by chromatography on silica gel (CH_2_Cl_2_) to afford the pure **3**.

*(E)-2-N-tert-Butyl-4-butylidene isoxazolidin-5-one* (**3a**): Yield: 60% as a viscous yellow oil; IR (neat) 1,760, 1,645 cm^-1^; ^1^H-NMR (δ ppm, *J* Hz): 6.68 (m, 1H), 4.00 (s, 2H), 2.14 (m, 2H), 1.49 (m, 2H), 1.17 (s, 9H), 0.97 (t, 3H, *J* = 7); ^13^C-NMR (δ ppm): 168.9 (*C*=O), 139.9 (=*C*H), 126.8 (=*C*), 59.9 (*C*(CH_3_)_3_), 49.7 (*C*H_2_-N), 32.3 (CH_2_), 24.4 (CH_3_), 21.4 (CH_2_), 13.8 (CH_3_); MS m/z (EI) 197 (M^+.^, 11), 182 (28), 141 (43), 57 (100), 56 (40), 44 (3), 41 (47), 29 (25); HRMS calcd. for C_11_H_19_NO_2_: 197.1416; found: 197.1407.

The article "An Expeditious Synthesis of [1,2]Isoxazolidin-5-ones and [1,2]Oxazin-6-ones from Functional Allyl Bromide Derivatives" was retracted in 2014. Reasons: misconduct by an author; duplicated images; duplicated data.

*(E)-4-Benzylidene-2-N-tert-butylisoxazolidin-5-one* (**3b**): Yield: 83% as a viscous yellow oil; IR (neat) 1,730, 1,595 cm^-1^; ^1^H-NMR (δ ppm): 7.53 (m, 5H), 7.52 (s, 1H), 3.36 (s, 2H), 1.22 (s, 9H); ^13^C-NMR (δ ppm): 170.2 (*C*=O), 140.3 (=*C*H), 135.4 (aromatic =*C*), 130.1 (aromatic =*C*H), 128.9 (aromatic =*C*H), 128.1 (=*C*), 124.6 (aromatic =*C*H), 60.4 (*C*(CH_3_)_3_), 40.2 (N*C*H_2_), 24.5 (*C*H_3_); MS m/z (EI) 231 (M^+.^, 14), 216 (24), 175 (49), 130 (48), 115 (64), 57 (100), 56 (45), 44 (4), 41 (53); HRMS calcd. for C_14_H_17_NO_2_: 231.1259; found: 231.1270.

*(E)-4-Butylidene-2-N-cyclohexylisoxazolidin-5-one* (**3c**): Yield: 48% as a viscous yellow oil; IR (neat) 1,725, 1,614 cm^-1^; ^1^H-NMR (δ ppm, *J* Hz): 6.68 (m, 1H), 3.40 (s, 2H), 2.73 (m, 1H), 2.17 (m, 2H), 1.96 (m, 10H), 1.27 (m, 2H), 0.96 (t, 3H, *J* = 7.00); ^13^C-NMR (δ ppm): 168.9 (*C*=O), 140.4 (=*C*H), 126.2 (=*C*), 67.8 (N*C*H), 54.7 (N*C*H_2_), 31.4 (*C*H_2_), 30.8 (*C*H_2_), 27.8 (*C*H_2_), 25.8 (*C*H_2_), 24.2 (*C*H_2_), 13.9 (*C*H_3_); MS m/z (EI) 150 (69), 136 (100), 94 (29), 82 (40), 80 (45), 67 (33), 56 (39), 55 (71), 53 (34), 44 (6), 41 (71); HRMS calcd. for C_13_H_21_NO_2_: 223.1572; found: 223.1583.

### 3.3. General procedure for the synthesis of methyl 2-alkyl-6-oxo-5,6-dihydro-2H-1,2-oxazine-4-carboxylates ***4***

*N*-Alkylhydroxylammonium chloride (31 mmol) and potassium *tert*-butoxide (30 mmol) in *tert*-butanol (45 mL) were placed in a 100 mL flask under a nitrogen atmosphere. The reaction mixture was stirred at reflux for 10 minutes then was added **2-*Z*** (10 mmol). After disappearance of the substrate (TLC), the solution was filtered under reduced pressure, evaporated and purified by chromatography on SiO_2_ with chloroform as an eluent to provide the pure **4**.

*Methyl 2-N-iso-propyl-6-oxo-5,6-dihydro-2H-1,2-oxazine-4-carboxylate* (**4a**): Yield: 79% as a yellow oil; IR (neat) 1,775, 1,730, 1,620 cm^-1^; ^1^H-NMR (δ ppm, *J* Hz): 8.04 (s, 1H), 4.01(m, 1H), 3.72 (s, 3H), 3.31 (s, 2H), 1.33 (d, 6H, *J* = 6.8); ^13^C-NMR (δ ppm): 171.1 (*C*=O), 170.5 (*C*=O), 149.0 (=*C*), 95.6 (=*C*H), 55.3 (*C*H(CH_3_)_2_), 51.8 (OCH_3_), 27.1 (NCH_2_), 19.4 (CH_3_); MS m/z (EI) 199 (M^+.^, 42), 168 (1), 157 (47), 125 (33), 98 (100); HRMS calcd. for C_9_H_13_NO_4_: 199.0845; found: 199.0855.

*Methyl 2-N-tert-butyl-6-oxo-5,6-dihydro-2H-1,2-oxazine-4-carboxylate* (**4b)**: Yield: 76% as a pale yellow oil; IR (neat) 1,778, 1,740, 1,660 cm^-1^; ^1^H-NMR (δ ppm): 7.90 (s, 1H), 3.54 (s, 3H), 3.13 (s, 2H), 1.22 (s, 9H); ^13^C-NMR (δ ppm): 170.9 (*C*=O), 170.5 (*C*=O), 147.4 (=*C*H), 95.8 (=*C*), 61.2 (*C*(CH_3_)_3_), 51.7 (O*C*H_3_), 27.1 (N*C*H_2_), 26.0 (*C*H_3_); MS m/z (EI) 213 (M^+.^, 5), 198 (1), 182 (47), 154 (3), 98 (6), 57 (100); HRMS calcd. for C_10_H_15_NO_4_: 213.1001; found: 213.1012. 

The article "An Expeditious Synthesis of [1,2]Isoxazolidin-5-ones and [1,2]Oxazin-6-ones from Functional Allyl Bromide Derivatives" was retracted in 2014. Reasons: misconduct by an author; duplicated images; duplicated data.

*Methyl 2-N-cyclohexyl-6-oxo-5,6-dihydro-2H-1,2-oxazine-4-carboxylate* (**4c**): Yield: 58% as a colorless oil; IR (neat) 1,757, 1,735, 1,624 cm^-1^; ^1^H-NMR (δ ppm): 8.03 (s, 1H), 3.72 (s, 3H), 3.30 (s, 2H), 2.02 (m, H), 1.53 (m, 10H); ^13^C-NMR (δ ppm): 170.9 (*C*=O), 170.7 (*C*=O), 148.2 (=*C*H), 94.4 (=*C*), 62.2 (N*C*H), 51.8 (O*C*H_3_), 29.7 (OC*C*H_2_), 27.2 (*C*H_2_), 24.8 (*C*H_2_), 24.2 (*C*H_2_); MS m/z (EI) 239 (M^+.^, 21), 180 (11), 126 (17), 83 (74). HRMS calcd. for C_12_H_17_NO_4_: 239.1158; found: 239.1170. 

## 4. Conclusions

We have developed a versatile synthetic approach to obtain [1,2]isoxazolidin-5-ones **3** in good yields and with total stereoselectivity. In addition, the method was used in the preparation of 4-functional heterocyclic compounds **4** in good overall yields. 
